The article "The Dialectic and Coupling of Three Paradigms in the Process of Art Rural Construction: Environment, Culture, and Industry" was retracted in 2023. Reasons: signs of a paper mill; suspected computer-generated content; unreliable results or conclusions; concerns about the data.

# The Dialectic and Coupling of Three Paradigms in the Process of Art Rural Construction: Environment, Culture, and Industry

**DOI:** 10.1155/2022/1864916

**Published:** 2022-08-03

**Authors:** Xiaoying Fan, Xianghu Zhong

**Affiliations:** ^1^School of Art, Southeast University, Nanjing 210000, Jiangsu, China; ^2^College of History and Culture, Hubei Normal University, Huangshi 435002, Hubei, China

## Abstract

The development and construction of cities and villages are a complex process jointly promoted by multiple subjects such as government, residents, enterprises, planners, and community elites. Through the summary and analysis of the practice of art rural construction at home and abroad, it is found that its events show three main paradigms in the development process. The environmental creation paradigm reconstructs the environmental semantics of the countryside through the creation of environmental art works, showing the remarkable characteristics of “the presence of works.” The cultural revival paradigm maintains the local culture through cooperation with residents in art and has the characteristics of “de-artization ” and “de-heritage.” The industrial development paradigm adjusts the industrial structure through the production of commodity art to achieve the improvement of the rural economic foundation. Under the new development trend, the three paradigms are gradually converging.

## 1. Introduction

Since the 1950s, art intervention in rural construction (referred to as “art village construction”) has gradually become a global cultural phenomenon. In the current art rural construction, artists intervene in rural construction in the form of art, so that “artists” can become the planners and implementers of rural construction and so that “art” can become a new resource of rural construction. Its goal is to activate rural culture, promote village revival, and rebuild the relationship between people and art, so as to explore various possibilities of rural revitalization, urban-rural integration, and village protection and development. And a large number of successful cases have emerged, such as the village of Akumedia in Italy; the village of Fiska in Finland; the village of Fiska in Poland; Salipa village, Echigo-Tsumari Area in Japan; and Gamcheon-dong village in Korea [1]. In the past decade or so, “artistic rural construction” has also become a common practice in China, and it has become an important way to revitalize the countryside with culture. Sex and other issues were discussed in depth, and a certain consensus was reached [2]. Nowadays, China is paying more and more attention to rural development. However, the development and construction of cities and villages are a complex process jointly promoted by the residents, enterprises, planners, community elites, and other subjects [3], as shown in Figure 1. The decline problem faced by rural areas in the process of urbanization has created many typical cases of art village construction and also achieved a boom in art village construction [4].

The article "The Dialectic and Coupling of Three Paradigms in the Process of Art Rural Construction: Environment, Culture, and Industry" was retracted in 2023. Reasons: signs of a paper mill; suspected computer-generated content; unreliable results or conclusions; concerns about the data.

Through the summary and analysis of the domestic and foreign art village construction practice, it is found that its events present three main paradigms in the development process [5] as shown in Table 1. The environmental creation paradigm reconstructs the environmental semantics of the countryside through the creation of environmental art works, showing the distinctive feature of “the presence of works”; the cultural revival paradigm maintains local culture through cooperative art with residents and has the characteristics of “de-artization” and “de-heritage” [6]. The industrial development paradigm adjusts the industrial structure through the production of commodity art and realizes the improvement of the rural economic foundation; the main construction content is as shown in Figure 1. Under the new development trend, the three paradigms are gradually moving toward integration [7].

Through the summary and analysis of the practice of art village construction at home and abroad, this paper compares and analyzes the characteristics of the three paradigms of art village construction and puts forward corresponding suggestions on the path selection of “art village construction.” This paper has great practical significance for promoting the construction and development of art village.

## 2. State of the Art

### 2.1. The Development Process of Art Village Construction

The early public art did not establish a connection with the countryside but appeared in cities, especially large cities, such as the cities that prevailed in the United States and European countries in the middle of the twentieth century, and then spread around the world [8]. In the new era of socialism with Chinese characteristics, China is committed to narrowing the gap between urban and rural dual structures and accelerating the pace of rural revitalization. Some artists have stationed themselves in the countryside and actively carried out art rural construction practice projects, which provide vivid practical cases for art to intervene in local creation and promote rural revitalization, but the research on the phenomenon of local creation in academia is relatively lagging behind. Due to the readjustment of the industrial structure in the new era, the loss of population in the process of urbanization, or the backward productivity and other problems, the social, economic, cultural, environmental, and other aspects of rural areas also have a relatively prominent decline [9]. Especially for countries where traditional farming culture has penetrated into the marrow of regional civilization, the development of public art in the new era has rapidly spread from cities to villages, becoming an important opportunity for rural revitalization [10]. In this new period, the development of public art pays more attention to the community, and the impact of art on rural development has become more diverse, complex, and profound. With the help of the rural turn of public art in objects and the anthropological turn in the way of thinking, the phenomenon of artists' involvement in rural construction has been very active in the past 20 years and even has the potential to form an art rural construction movement [11].

The article "The Dialectic and Coupling of Three Paradigms in the Process of Art Rural Construction: Environment, Culture, and Industry" was retracted in 2023. Reasons: signs of a paper mill; suspected computer-generated content; unreliable results or conclusions; concerns about the data.

The practice of art village construction does not happen overnight, and it has shown a certain continuity and development around the world [12]. The mountain village of Valloria, on Italy's Mediterranean coast, faced hollow decay in the 1990s due to population loss [13]. Several returning young people spontaneously set up an organization named after the famous local scenic spot “Three Springs,” put forward the idea of “Opening Your Heart,” and invited artists to use the door panels of every household in Valloria as canvases to create [14]. The strong creative atmosphere quickly stimulated the exhibition and sales of a number of cultural and creative products such as ceramic glass products, textile design, and jewelry design. Under the influence of artists, the government decided to build Bornholm into a center for handicrafts, promote the establishment of the Arts and Crafts Association Bornholm (ACAB), organize international handicraft exhibitions, and supervise the quality of handicraft products, making them integrated with the local tourism industry [15].

Influenced by the long and heavy agricultural civilization, there are more practical cases of art village construction in Asia [16], as shown in Table 2. As a result, agricultural productivity was greatly reduced, and private houses and schools were once vacant [17]. By holding the art festival, the local area has realized the transformation from the traditional agriculture to the cultural tourism industry and has also set up a demonstration of “artistic revitalization of the countryside” in the world [18]. In South Korea, in the middle of the last century, immigrants from civil war gathered in Gamcheon-dong and built a large number of shantytowns. Since the 1980s, due to the deterioration of living conditions and architectural style, Gamcheon-dong has been left with the impression of a chaotic and backward area [19]. In 2012, Tugou village put forward the construction goal of “Rural Art Museum,” treating the entire village as an open-air art museum to build, from point (art collection display), line (“village house art exhibition” connecting settlements), and surface (Earth art of idyllic sowing), three dimensions to realize the artization of rural environment, as shown in Figure 2.

The article "The Dialectic and Coupling of Three Paradigms in the Process of Art Rural Construction: Environment, Culture, and Industry" was retracted in 2023. Reasons: signs of a paper mill; suspected computer-generated content; unreliable results or conclusions; concerns about the data.

Yin Aimu listed many rural art intervention projects since the 21st century and proposed that the construction of art townships should combine local characteristics and develop rural industries. Li Qin analyzed the case of art intervention in rural construction in Yuanyang, Yunnan province, and believed that the creation of “Haneva” in the process of Yuanyang art township construction reflects the local nature of art intervention, so it can stimulate the emotions of villagers and gain their recognition. In most regions, art township is playing an increasingly important role in exploring China's new urbanization and urban-rural relations.

## 3. Method

### 3.1. Path Selection of “Art Village Construction”

The forms and media of art intervention in rural construction need to be adapted to local conditions, and the methods used for different terrains, cultural backgrounds, and customs are different. It should be closely combined with the actual needs and actual conditions of local residents, and appropriate forms of intervention should be chosen according to local conditions to achieve the purpose of art to help rural revitalization. Meng Fanxing and Kang Zenan proposed that there are three main paths for art to intervene in rural construction, namely, cultural protection, landscape reconstruction and space production, and subjectivity reshaping. This is specifically shown in Figure 3. Xurui also summarizes three paths: one is to hold large-scale art festivals, the second is to restore the social and cultural ecology, and the third is to attract urban people to settle in the countryside and build them together [20].

The first path of “artistic village construction” is to hold large-scale art festivals. The “Xucun Plan” and the “Qingtian paradigm” proposed later have explored extremely valuable experiences in the construction of China's rural art culture. Xucun is a remote mountain village in Heshun county, Shanxi province, where the artist Qu Yan has been stationed for ten years. Through the early investigation of the history and culture, customs and habits, and terrain and landforms of Xu village, he gradually sorted out the “Xu Village Plan” into shape. The worship of land gods is popular in the Xucun area, so Qu Yan held the first Xucun International Arts Festival in 2011 with elements such as the “Stove Fire Festival” and the Land Temple as the starting point to preserve and revive folk customs. The second edition of the festival was named after “Return of the Soul” and aimed to inherit the culture of the local ancestral hall. So far, the Xucun International Arts Festival has been successfully held five times.

The article "The Dialectic and Coupling of Three Paradigms in the Process of Art Rural Construction: Environment, Culture, and Industry" was retracted in 2023. Reasons: signs of a paper mill; suspected computer-generated content; unreliable results or conclusions; concerns about the data.

The second path of “artistic rural construction” emphasizes the overall restoration of rural society and cultural ecology. Its basic strategy is to “dress and cap” the houses of the entire village first and then hold various curatorial events, including art festivals, rather than to mainly focus on art festivals. This model often pays more attention to local traditional handicrafts. Because, in order to restore the local social and cultural ecology, the economic aspect is the most important. After four or five years of this activity, it was declared a failure. Although the “Bishan Project” was unsuccessful, it had a great influence, especially as an idea of “artistic village construction,” which was representative. Later, when reflecting on his “art township building” road, Qu Yan basically denied his mode of “art township building” in Xucun but tended to the “Bishan Plan” mode made by Ou Oning and Zuo Jing and then put forward the “Qingtian paradigm.” As shown in Figure 4, the so-called “Qingtian paradigm” means to use local traditions from history, economy, belief, etiquette, nature, environment, agriculture, and folk life; then to form new cultural values and social ecology; and then rebuild the rural community society. The “Qingtian paradigm” does not seem to highlight the artistic and aesthetic factors, so why do we still say that it is an “art hometown construction”? Mainly because artists play a leading role in it. The “Qingtian paradigm” still has a great influence among the artists or other intellectuals engaged in the “art township building” all over the country.

The third path of “artistic rural construction” is to attract urbanites to go to the countryside to settle down and build together. The core issue of rural revitalization and rural development is the issue of talents and manpower. It is not a shortage of people in the countryside, but a shortage of young adults and talents, which is a structural shortage. So how to solve this problem? Undoubtedly, attracting talents and manpower back to the countryside is the key. However, the return of talents may encounter some policy obstacles, cognitive obstacles, and other problems at present. Only some places with special endowments can realize the return of talents and manpower to the countryside.

The article "The Dialectic and Coupling of Three Paradigms in the Process of Art Rural Construction: Environment, Culture, and Industry" was retracted in 2023. Reasons: signs of a paper mill; suspected computer-generated content; unreliable results or conclusions; concerns about the data.

### 3.2. The Aesthetic Illusion of “Artistic Village Construction”

In the practice of “artistic village construction,” the aesthetic concept of artists is often not recognized by the villagers. Sun Jun recalled, “When I first entered the village, I joined the village renovation and improvement work as an artist. I hoped to use art to activate the village. I liked the works I created during this period, and my teachers and colleagues also highly praised them. But the villagers at that time did not like these works at all. For more than 100 years, the government and intellectuals have implanted a modern aesthetic concept in the hearts of the villagers, that is, only new, useful and urban are beautiful, and the local old, traditional means backward.

At present, China's art intervenes in the practice of local creation, and the transformation or reconstruction of some rural buildings, spaces, and environmental landscapes ignores the cultural characteristics of local customs. Migrant workers and local villagers are influenced by the concepts of urban modernization, urban landscape, aesthetic standards, etc. and also tend to rebuild the original village greening, housing construction, public space, etc. according to urbanization standards, so the overall artistic aesthetic and landscape transformation of the countryside have a homogeneous tendency. Rural construction seems to have entered the strange circle of imitation and replication, the successful experience of rural construction in a place seems to have become a standardized template for “beautiful villages,” and the tendency of art township construction is to be formatted, patterned, and uniformized, while ignoring localization, personalization, and differentiation; the consequence of this phenomenon is the lack of staying power of local creation.

## 4. Results and Analysis

### 4.1. The Paradigm of Environmental Construction in Art Village Construction

Generalized environmental art including architectural art, garden art, and outdoor installation art is the main direction for artists to carry out rural art practice, as shown in Figure 5.

The artist's artistic realization of the rural environment through the creation of works is the most intuitive expression of the environment creation paradigm. Therefore, the “presence of the work” has naturally become the most prominent feature of this paradigm at the phenomenal level. Different from traditional art forms such as painting, music, and literature, environmental art works generally have the closest relationship with the subject of their appreciation. The first contact between the subject and the countryside is the environment, and the artistic transformation of the rural environment prompts the subject to have a strong sense of artistic presence in the process of perception and experience. Compared with the lively scene of the continuous production of art exhibition space, the relationship between local villagers and works of art is worrying. Although art works attract foreign artists and tourists, they are rarely directly related to the lives of villagers. This makes one wonders, do the villages really need art galleries? Its purpose is to break the boundaries between urban and rural areas and gradually realize the social justice of aesthetics. Although the phenomenon of artistic intervention at this stage is often misunderstood as the wishful thinking of the artist, in the long run, its influence on the aesthetic consciousness of the villagers should be positive and subtle. Through the influence on the villagers' aesthetic consciousness, they can find the artistic meaning of the artistic creation environment and integrate the art into their lives, so as to shorten the distance between them and the art.

The article "The Dialectic and Coupling of Three Paradigms in the Process of Art Rural Construction: Environment, Culture, and Industry" was retracted in 2023. Reasons: signs of a paper mill; suspected computer-generated content; unreliable results or conclusions; concerns about the data.

### 4.2. The Cultural Revival Paradigm of Art Village Construction

Art intervention in rural construction should be rooted in the local natural environment and cultural characteristics and comprehensively consider the overall environment and local characteristics of the countryside. In recent years, the rural transformation in some places has shown a trend of “local-space tension,” and some villages have blindly copied and imitated in the process of planning and construction, not according to the actual situation of the countryside, resulting in the scene of “one side of a thousand villages.” In the artistic process of rural environment, some artists have done critical thinking on the above-mentioned environment creation paradigm and believed that art rural construction should not be wasted directly in the figurative process of artistic creation, but from the perspective of art ontology do some reflection. The problems faced by most rural areas in China are the decline of environmental quality and the decline of local culture. However, the phenomenon of farmers “leaving the soil” caused by urbanization has brought unprecedented pressure to the inheritance and development of rural culture. The urgent problem of rural construction is not only the renewal of the material landscape and the cultivation of the industrial economy, but also how to promote the social development of rural communities by revitalizing the local culture that has been gradually disintegrating under the influence of globalization and urbanization. So, artists began to call that “art village construction” and “art village construction” are not the same thing. Artists should proceed from the standpoint of respecting local knowledge, no longer confined to the traditional category of “art creation,” and directly take the social practice of rural construction as a creative process. The “cultural revival paradigm” was born from this.

The article "The Dialectic and Coupling of Three Paradigms in the Process of Art Rural Construction: Environment, Culture, and Industry" was retracted in 2023. Reasons: signs of a paper mill; suspected computer-generated content; unreliable results or conclusions; concerns about the data.

In general, the cultural revival paradigm is devoted to the excavation and inheritance of local culture and respects the authenticity of culture. However, based on this basic law, the paradigm further criticizes and reflects on the current general art village construction, material, and intangible cultural heritage protection and further reflects the transformation of the following two dimensions.

#### 4.2.1. “De-artization” of Intervention Methods

Under the influence of successful cases, a large number of artists began to go to rural areas, and the creation of works such as land art, architecture, sculpture, and murals with rural themes began to become the origin of art intervention in rural construction. However, due to the lack of long-term accumulation and practical experience of rural life and field investigations that go deep into local society and history, a large number of works cannot be closely related to rural life and local context but simply depict different artists' personal views of “field idyll-style utopia.” These social practices themselves do not have the characteristics of art but stand in the position of authenticity of local culture, showing tendencies such as sociology or anthropology.

#### 4.2.2. “De-heritage” of Work Policy

Although the revival of culture always revolves around the authenticity of local culture, the artist is not and does not want to be a heritage protection worker. Whether it is a material form of heritage or an intangible form of heritage, the focus of the artist's work is not through ancient buildings. The means of repairing and inheriting skills is not to “reproduce” the heritage but to bring the heritage back to life. The disappearance of local traditional architecture and craftsmanship is the result of the failure of local culture to adapt to the new way of life in the context of globalization and urbanization. This means that the “evolution” of local culture requires sacrificing a part of its authenticity to maintain its cultural vitality, and the artist's job is to try to minimize the loss of this authenticity.

### 4.3. The Industrial Development Paradigm of Art Village Construction

The industrial development paradigm is that artists intervene in the industrial construction of the countryside to promote the revitalization of the rural economy. In the process of rural construction, it generally follows the laws of industrial economics from a gathering area formed spontaneously by artists to an art industrial park. In order to improve their professional skills, promote their works and meet more artists, curators, critics, and even future employers. The village of Montmartre in the north of Paris, France, was originally just a remote and low-cost village, attracting a large number of painters, sculptors, writers, musicians, architects, and interns who were struggling to make ends meet. With the gathering of artists, a large number of exhibition halls, galleries, and art dealers have gradually settled in, making the village itself undergo earth-shaking changes and become a well-known art highland today.

The article "The Dialectic and Coupling of Three Paradigms in the Process of Art Rural Construction: Environment, Culture, and Industry" was retracted in 2023. Reasons: signs of a paper mill; suspected computer-generated content; unreliable results or conclusions; concerns about the data.

Although the main purpose of the gathering of young artists is to seek their own development with no intention of intervening in rural construction, the presence of artists has injected new vitality into the isolated and backward rural communities. More importantly, artists create, communicate, and exhibit in the countryside, attracting art dealers and tourists, and potential markets are quietly born, laying the foundation for the development of the traditional art industry and even today's cultural and creative industry.

Among the many industry-led art villages in China, Shenzhen's Dafen oil painting village has become China's most famous art industrial park relying on the countryside with its output value of hundreds of millions. In 1989, Hong Kong painter and art dealer Huang Jiang came to Shenzhen to copy and sell oil paintings. He settled in Dafen village because of the cheap rent advantage and started to produce line paintings, which were specially supplied to Walmart supermarkets in the United States. With the development of export trade, the demand for line paintings has increased, production has gradually turned to streamlined production, and the number of painters employed has also increased. Under the influence of the development trend and law of the industrial economy with creativity as the core, most art villages have shifted from single-form commodity art production and sales villages to comprehensive cultural and creative industrial parks in terms of development path and industrial structure.

In the industrial development paradigm, although the intervention of artists may not be entirely for commercial purposes, it is mainly “commodity art” and accompanying industries such as tourism that promote the development of rural economy. Of course, in real cases, regardless of environmental creation or cultural revival, most villages have realized the development of industries, especially tourism industries, after the intervention of artists.

The article "The Dialectic and Coupling of Three Paradigms in the Process of Art Rural Construction: Environment, Culture, and Industry" was retracted in 2023. Reasons: signs of a paper mill; suspected computer-generated content; unreliable results or conclusions; concerns about the data.

### 4.4. The Core of Art Village Construction: Environment, Culture, and Industry

At the practical level, the three paradigms of environmental creation, cultural revival, and industrial development appeal to the different starting points chosen by artists when carrying out rural construction activities. Industry, these three cores appeal to three important problems faced by rural areas in our country.

In terms of environment, from the end of the last century to the beginning of this century, the large-scale evacuation of villages and relocations caused constructive damage to the original rural living environment, and traditional buildings and street spaces were destroyed. Under the influence of globalization and urbanization, villagers took the opportunity of improving production and living conditions to redefine their home landscape by using materials such as concrete and color steel tiles, breaking the local order of the original environment.

In terms of culture, the dissemination of information and value changes as internal factors and the changes of population structure, society, and natural environment as external factors have jointly caused the variation of rural culture. The improvement of traffic conditions and the development of new media technologies have made the exchange of information between rural areas and urban areas more frequent. Urban thinking and urban lifestyles have impacted local culture, and cultural events and cultural ceremonies such as festivals, customs, beliefs, and clan relations have faced challenges, difficult choice of alienation or decline.

In terms of industry, although the country's economic aggregate is expanding, the added value of the primary industry has gradually declined in the past 15 years. The “local Chinese society” is no longer economically dependent on the primary industry. The situation is as follows: Industrial development in rural areas has created enormous pressure. The second and tertiary industries continue to erode the traditional agriculture, forestry, animal husbandry, and fishing, and the resolute adjustment of the rural industrial structure has made the countryside lose its foundation and transformed it into some other kinds, in the sense of production areas, parks, scenic spots, and even business districts.

Based on the above three aspects, the three paradigms of art intervention give different responses. The intention of the environmental construction paradigm is to promote the renewal of rural landscapes through broad environmental art design, and the renewal process is not only to promote the metabolism of rural landscapes, but also to introduce artistic and creative construction thinking, in order to improve the rural ecological environment and the quality of human settlements. At the same time, the environment is regarded as a work to be displayed to attract visitors. The cultural renaissance paradigm aims to uphold the principle of authenticity to revitalize local culture. Its intervention method is influenced by anthropology and sociology. It advocates uniting local residents, removing the main role of artists, and regards the process of mutual assistance as the formal composition of works, which is a contemporary. In this context, efforts have been made to maintain the rural society. The industrial development paradigm follows the development path from the artist gathering area to the art industrial park, develops the art industry through the production of commodity art, gradually replaces the primary industry in the industrial structure, creates capital under the guidance of the law of market operation, and provides rural areas, guarantee of economic development. The comparison of the three intervention paradigms is shown in Table 3.

The article "The Dialectic and Coupling of Three Paradigms in the Process of Art Rural Construction: Environment, Culture, and Industry" was retracted in 2023. Reasons: signs of a paper mill; suspected computer-generated content; unreliable results or conclusions; concerns about the data.

It needs to be emphasized that the three intervention paradigms only represent the different starting points or emphases selected by the artists in the rural construction action based on their own knowledge background and combined with the actual situation of the case. This does not mean that the three paradigms are limited to solving their corresponding rural problems. In fact, with the continuous deepening of the artist's rural construction practice, environmental, cultural, and industrial problems have also been exposed. When implementing the rural construction plan, the artist also hopes to jointly realize the comprehensive revitalization of the case village from three aspects. From Echigo-Tsumari in Japan to Changtangzi village in Yunnan, China, the creation of rural environmental art has never been purely environmental transformation. The creation of works and the planning of exhibitions have taken into account the development of the accompanying tourism industry. From the left Jing and Ou Ning's Bishan Plan to Qu Yan's Xucun Declaration, the rural cultural revival plan formulated by the artist also always includes the restoration and reuse of vernacular architecture, residential courtyards, public spaces, and other living environments. From Fen to Songzhuang in the north, the creation of the art industry highland is more connected with the reconstruction and promotion of local culture.

Recently, the art village construction team represented by the curator Zuo Jing put forward the theory of “three productions” after summarizing the previous practical experience in Anhui, Guizhou, and Yunnan: the production of space, the production of culture, and the production of products. The core of the three art villages of environment, culture, and industry has been unified and sorted out. At the end of 2016, Zuo Jing's team came to Wengji village in Jingmai mountain, Yunnan province, to solve rural environmental, cultural, and industrial problems in parallel and started the “Jingmai Mountain Project” after a detailed inspection of the local natural ecology and human ecology. In terms of environmental renovation, the artists carried out repairs to some of the traditional dry-column buildings in the Wengji Bulang ancient village and gave the building space new vitality with exhibition halls and homestays; in terms of cultural revival, the artists collected and sorted out the historical context of the village and reproduced it as a “local teaching material” through text, hand-painting, and multimedia, providing a way for residents, especially children, to reunderstand the village culture; the work in industrial construction combines cultural revival and environmental transformation. Tea culture: the interpretation of the hotel and the creation of homestays help the integrated development of the local tea economy and tourism industry. It can be seen that against the background of the anthropological turn of the artist's thoughts on rural construction and the commercialization of rural construction activities, several types of construction paradigms formed in the early stage are gradually disappearing into each other.

The article "The Dialectic and Coupling of Three Paradigms in the Process of Art Rural Construction: Environment, Culture, and Industry" was retracted in 2023. Reasons: signs of a paper mill; suspected computer-generated content; unreliable results or conclusions; concerns about the data.

Nowadays, the ideological trend of “social restoration” in rural areas promotes “artistic rural construction” to break through the stubbornness of the paradigm step by step. The reconstruction of environmental semantics, the transformation of culture and art, and the transformation of industrial structure have become the common focus of artists' intervention. “Art village construction” is developing in the direction of originating from the field of art but beyond the field of art. Under the guidance of the top-level design of Beautiful China and Beautiful Countryside, the aesthetic value of socialism with Chinese characteristics in the new era has returned to the standard of rural construction, providing more opportunities for the active display of the artist's aesthetic knowledge structure and social practice ability. At the same time, national policies and theoretical and practical development trends have promoted the path innovation of art rural construction, making it gradually enter a new historical stage, bringing a richer and more prosperous future to China's rural construction.

## 5. Conclusion

As we all know, “rural revitalization” is a national strategy. How to achieve rural revitalization requires a lot of exploration. The integration of art into rural construction and art and rural modernization construction is a new strategy for transforming rural landscapes, beautifying rural cultural spaces, defending rural characteristic culture, and promoting rural revitalization in the context of local creation, and “art village construction” can not only bring tangible benefits to rural areas in terms of material production, rural tourism, investment attraction, etc., but also promote the restoration of rural internal culture, so that the village embarks on a virtuous circle of self-development. In this regard, “art village construction” provides a very effective landing path for rural revitalization. Art intervention in rural construction should take local villagers as the main body of rural construction, hook local historical and cultural resources, do a good job of local culture filing, take the construction of public art in visual form and integrate it into local life art projects as the theme to form regional characteristic work content, take the revitalization of local culture as the goal, combine the cultural tourism industry, promote rural aesthetic education actions, restore the innovative vitality of rural areas, and promote the growth of local traditional culture, so as to create a sustainable cultural format for rural revitalization.

The article "The Dialectic and Coupling of Three Paradigms in the Process of Art Rural Construction: Environment, Culture, and Industry" was retracted in 2023. Reasons: signs of a paper mill; suspected computer-generated content; unreliable results or conclusions; concerns about the data.

## Figures and Tables

**Figure 1:** The construction framework of the art township construction.

**Figure 2:** Three dimensions of the art township construction of Tugou village.

**Figure 3:** Three paths for art township construction.

**Figure 4:** The content of the Qingtian paradigm.

**Figure 5:** The main directions for artists to carry out rural art practice.

**Table 1:** Comparison of the characteristics of the three main paradigms of art village construction.

Type	Environment creation paradigm	Cultural revival paradigm	Industrial development paradigm
Features	“Presence of works”	“De-artization,” “de-heritage”	Adjusting the industrial structure through the production of commodity art, and realizing the improvement of the rural economic foundation

**Table 2:** Practical cases of art village construction in Asia.

	Paradigm of environment construction	Paradigm of cultural revival	Paradigm of industrial development
Typical cases	Echigo-Tsumari area in Japan, Gamcheon-dong village in Busan, South Korea, Shijiezi village in Tianshui, Gansu, Fuyang Wen village in Hangzhou, Changtangzi village in Maitreya in Yunnan, Bishan village in Yi county	Anhui province; Heshunxu village in Shanxi province; Qingtan township in Xiangtan town, Foshan; Tiancun, Guangdong; Wushan town, Xiangyang, Hubei; Haotang village, Xinyang, Henan	Montmartre village, Paris, France; Greenwich village, New York; Dafen village, Shenzhen, Guangdong; Xiaobao village, Songzhuang, Tongzhou, Beijing

The article "The Dialectic and Coupling of Three Paradigms in the Process of Art Rural Construction: Environment, Culture, and Industry" was retracted in 2023. Reasons: signs of a paper mill; suspected computer-generated content; unreliable results or conclusions; concerns about the data.

**Table 3:** Comparison of three art village construction paradigms.

	Paradigm of environment construction	Paradigm of cultural revival	Paradigm of industrial development
Art form	Environmental art	Collaborative art	Commodity art
Process characteristics	Independent creation	Joint local residents	Cluster production
Effectiveness of intervention	Subjectivization/production	Desubjectivization	Productization
Intervention goal	Reconstruction of environmental semantics	Inheritance and interpretation of local culture	Replacement of art industry
Spatial attributes	Transformation of connotation-production of display space	Continuation of connotation	Transformation of connotation-production of consumption space
Existing problems	Local context breakage	Only social and ethical standards	Consumerist aesthetics and low participation of residents

## Data Availability

The dataset used to support the findings of this study is available from the corresponding author upon request.
